# Natural Compounds for SIRT1-Mediated Oxidative Stress and Neuroinflammation in Stroke: A Potential Therapeutic Target in the Future

**DOI:** 10.1155/2022/1949718

**Published:** 2022-09-05

**Authors:** Chaoyou Fang, Houshi Xu, Ling Yuan, Zhengyang Zhu, Xiaoyu Wang, Yibo Liu, Anke Zhang, Anwen Shao, Meiqing Lou

**Affiliations:** ^1^Department of Neurosurgery, Shanghai General Hospital, School of Medicine, Shanghai Jiao Tong University, Shanghai, China; ^2^School of Public Health, Shanghai Jiaotong University School of Medicine, Shanghai, China; ^3^Department of Neurosurgery, The Second Affiliated Hospital, School of Medicine, Zhejiang University, China; ^4^Clinical Research Center for Neurological Diseases of Zhejiang Province, Hangzhou, China

## Abstract

Stroke is a fatal cerebral vascular disease with a high mortality rate and substantial economic and social costs. ROS production and neuroinflammation have been implicated in both hemorrhagic and ischemic stroke and have the most critical effects on subsequent brain injury. SIRT1, a member of the sirtuin family, plays a crucial role in modulating a wide range of physiological processes, including apoptosis, DNA repair, inflammatory response, and oxidative stress. Targeting SIRT1 to reduce ROS and neuroinflammation might represent an emerging therapeutic target for stroke. Therefore, we conducted the present review to summarize the mechanisms of SIRT1-mediated oxidative stress and neuroinflammation in stroke. In addition, we provide a comprehensive introduction to the effect of compounds and natural drugs on SIRT1 signaling related to oxidative stress and neuroinflammation in stroke. We believe that our work will be helpful to further understand the critical role of the SIRT1 signaling pathway and will provide novel therapeutic potential for stroke treatment.

## 1. Introduction

Stroke is a type of fatal cerebral vascular disease with a high mortality rate [1], the second leading cause of death, and the leading cause of disability worldwide [2, 3]. As a result of stroke, a substantial economic and social burden is imposed [4]. Stroke can be classified as either an ischemic stroke or a hemorrhagic stroke [5, 6]. Furthermore, hemorrhagic stroke may be divided into intracerebral hemorrhages (ICHs) and subarachnoid hemorrhages (SAHs). In the event of hemorrhage and ischemia, overproduction of reactive oxygen species (ROS) and neuroinflammation have been linked to subsequent brain injury [7, 8, 9]. ROS overproduction is closely related to neuroinflammation, with each promoting and amplifying the other. After a stroke, mitochondria overproduce ROS, which then causes a wide array of destructive effects on cellular functions by damaging proteins, lipids, and nucleic acids [10, 11, 12, 13]. In addition, cell death pathways can be signaled by ROS as intracellular messengers [14]. Additionally, microglia and astrocytes are activated within hours of a stroke, releasing cytokines and chemokines in addition to leukocyte infiltration [15, 16, 17]. Reducing ROS and neuroinflammation has long been a focus of stroke treatment research. New therapies that reduce oxidative damage and inflammation after stroke could improve neurological recovery.

Silent mating type information regulation 2 homolog 1 (SIRT1), also known as sirtuin 1, is an NAD-dependent deacetylase located in the nucleus [18]. SIRT1 has been proven to play a critical role in modulating a wide range of physiological processes, including apoptosis, DNA repair, inflammatory response, metabolism, cancer, and stress [19, 20]. Previous studies have demonstrated that SIRT1 can protect against oxidative stress and inflammation in various research areas, including ischemic reperfusion-induced renal, brain, and heart injuries [21, 22, 23]. In recent years, SIRT1 has been recognized as particularly important in the pathogenesis of stroke [24, 25, 26]. SIRT1 modulates oxidative stress and inflammation through a variety of signaling pathways. Numerous studies have demonstrated that SIRT1 can protect neurons against oxidative and inflammatory damage induced by FOXOs, nuclear factor-*κ*B (NF-*κ*B), and p53 [25, 27, 28]. Reducing ROS and neuroinflammation by targeting SIRT1 may represent a promising therapeutic target for stroke.

During ischemic stroke, brain tissue is hypoxic due to vascular obstruction. The only FDA-approved treatment for ischemic stroke is tissue plasminogen activator (tPA) [29]. However, the limited therapeutic window of this drug is a major concern, as it can cause secondary damage that is ischemia–reperfusion injury [30, 31]. Despite significant progress in the clinical treatment of the disease, there has not been a medical or surgical therapy to improve outcomes for patients with hemorrhagic stroke. Surgical intervention in hemorrhagic strokes is still controversial. As a result, it is crucial to define the pathogenesis and targets for the prevention and treatment of stroke. In addition, we discuss the potential mechanisms and natural compounds used for stroke treatment by which SIRT1 protects against stroke through antioxidative and anti-inflammatory effects.

The following search terms were used: SIRT1, oxidation, neuroinflammation, and stroke. Once we found the target article, we continued our search in the similar articles section of PubMed. Then, we screened studies in English that investigated interventions for natural compounds in stroke. This review summarized the potential mechanisms and natural products used in stroke by which Sirt1 protects against stroke through antioxidative and anti-inflammatory effects.

## 2. Activation Mechanism

### 2.1. SIRT1-Mediated Antioxidation in Stroke

ROS are a class of oxygen-containing reactive chemicals that play essential roles in normal physiological processes, for instance, in controlling redox regulation of protein phosphorylation, ion channels, and transcription factors [32]. Typically, the primary intracellular source of ROS in mammalian cells is thought to be mitochondria [33, 34]. However, a high concentration of ROS can cause irreversible changes in protein, lipid, carbohydrate, and nucleic acid structures [35]. ROS has been proved to play a vital role in developing neuronal damage after a stroke [36, 37].

During ischemic injury, oxidative stress is one of the earliest outcomes, causing cascades of cellular and molecular processes that cause neurodegeneration and death of neurons [38]. Increased levels of ROS in cells, such as hydroxyl radicals, can result in oxidative stress and mitochondrial dysfunction, which can lead to cerebral ischemia and further aggravate the cerebral injury [39, 40].

SIRT1 is the most extensively studied sirtuin and is expressed in the brain at a higher level than other organs [41]. According to a previous study, mice overexpressing SIRT1 sustained less hippocampal damage following cerebral ischemia (bilateral common carotid artery occlusion) than mice lacking SIRT1, demonstrating that SIRT1 plays a prominent role in brain protection [42]. In addition, SIRT1 has been identified as playing an essential role in oxidative stress [41, 43]. SIRT1 is activated after the onset of stroke and can regulate multiple signaling pathways to affect oxidative stress, further regulating the pathological process of stroke. This section summarizes the critical signaling pathway proteins in the process of SIRT1-mediated antioxidation in stroke. The signaling pathway of SIRT1-mediated antioxidation in stroke is shown in Figure 1.

#### 2.1.1. PGC-1*α*

According to previous research, peroxisome proliferator-activated receptor gamma coactivator 1-*α* (PGC-1*α*) functions as a master regulator of mitochondrial function and biogenesis, such as oxidative phosphorylation (OXPHOS) and ROS detoxification, contributing to maintaining metabolic homeostasis [44]. The expression of PGC-1*α* is high in tissues with active oxidative metabolism, especially in the brain [45]. PGC1-*α*, mainly by upregulating oxidation defense, is critical in preventing cell death due to mitochondrial dysfunction [46]. To prevent oxidative stress-induced cell damage, the expression of PGC-1*α* is positively regulated by oxidative stress [47]. In addition to exerting a pivotal role in preventing oxidative damage, the upregulation of PGC-1*α*-antioxidant target genes also significantly decreased mitochondrial ROS levels and ensured mitochondrial integrity [48]. Synthesizing ATP in mitochondria inevitably leads to electrons leaking into oxygen, which eventually results in ROS formation [49]. By activating several transcription factors, including NRF, Tfam, ERR*α*, and PPARs, PGC-1*α* increases mitochondrial biogenesis and the function of genes [50]. Additionally, PGC-1*α* is involved in regulating mitochondrial antioxidant defenses. Manganese superoxide dismutase (MnSOD/SOD2), peroxiredoxin (Prx) 5, Prx3, thioredoxin reductase (TRXR) 2, UCP-2, thioredoxin (TRX) 2, and catalase are increased by PGC-1*α* and consequently prevent mitochondrial dysfunction in cells [46]. An increase in PGC-1*α* expression is related to preventing oxidative damage by cells when exposed to oxidative stress [47]. Mouse experiments confirmed that mice lacking PGC-1*α* are more susceptible to oxidative damage [51].

Regulation of PGC-1*α* occurs at the transcriptional and posttranslational levels. The significant transcription factors are FoxO1 and FoxO3, which regulate the expression of the PGC-1*α* gene in a tissue-dependent way [52]. More importantly, PGC-1*α*, a downstream effector of SIRT1, plays a neuroprotective role [53]. Numerous studies have shown that when SIRT1 is activated, it can deacetylate downstream PGC-1*α*, which exerts antioxidative and anti-inflammatory effects [53, 54]. As one of the targets of SIRT1, PGC-1*α* suppresses ROS production by inducing ROS detoxifying enzymes [55]. Thus, neurons are substantially protected against oxidative stress by increasing SIRT1-mediated PGC-1*α* levels [55]. The NAD+/NADH ratio measures the redox state of cells [56]. As NAD+/NADH levels rise, SIRT1 becomes activated, deacetylating PGC-1*α* [57].

An experimental study based on a cerebral ischemia model showed that SIRT1, FOXO1, PGC-1*α*, Bax, and Bcl-2 protein expressions were significantly reduced after oxygen-glucose deprivation/reperfusion (OGD/R) [58]. Calycosin-7-O-*β*-D-glucoside (CG), a representative drug, downregulated the expression of Bax, which further suggests that CG protects against ischemic stroke by activating the SIRT1/FOXO1/PGC-1*α* signaling pathway. In addition, many other drugs have been shown to exert neuroprotective effects by upregulating SIRT1-dependent PGC-1*α* expression to induce antioxidation in stroke. In previous studies, SIRT1/PGC-1*α* signaling was shown to enhance SOD levels, remove MDA from the cell, and decrease oxidative stress, leading to cell death resistance [59].

#### 2.1.2. Forkhead Transcription Factors of the O Class (FOXO)

The mammalian FOXO have four members, including FOXO1, FOXO3, FOXO4, and FOXO6 [60]. Several processes in the body are controlled by FOXO, including the cell cycle, metabolism, stress resistance, and inflammation [61, 62]. Among them, FOXO3 has been demonstrated to play an essential role in the regulation of oxidative stress, which can upregulate the expression of several antioxidant proteins, including superoxide dismutase (SOD), manganese superoxide dismutase (MnSOD), and catalase (CAT) [63, 64, 65, 66]. FOXO3 can be phosphorylated and deacetylated to regulate its transcriptional activity [67].

In addition, it has been shown that SIRT1 deacetylates histone and nonhistone proteins, including FOXO [68]. SIRT1 increases cellular resistance against oxidative stress by deacetylating and activating FOXO, which promotes the expression of antioxidant proteins such as SOD [69]. Deacetylation of FOXO3 by SIRT1 can prevent cell death induced by FOXO3 [69]. In response to stimulation, FOXO3a phosphorylates and binds to 14-3-3 proteins in the nucleus. This inhibits FOXO3a-dependent transcription [70]. Cells can resist oxidative stress and induce cycle arrest by deacetylating FOXO3 with SIRT1. Wu et al. found that the lncRNA SNHG12 inhibits the oxidative stress response of the ischemia/reperfusion (I/R) model by activating the SIRT1/FOXO3 pathway [71]. PGC-1*α* transcription is also regulated by FoxO transcription factors in different cell types. The FoxO3 signaling molecule interacts directly with PGC-1*α* in vascular endothelial cells and protects mitochondria from oxidative stress through a mechanism controlled by activation of SIRT1 [72]. When FoxO3 is inactivated and PGC-1*α* is downregulated, ROS detoxification is hampered [73]. FoxO3 can be inactivated by the PI3K/Akt signaling pathway to further decrease endothelial PGC-1*α* expression [69]. In the research of Duan et al., Akt/SIRT1/FOXO3a/PGC-1*α* pathways are shown to be regulated by saponin from Aralia taibaiensis (sAT), protecting brain cells from ischemia and reperfusion- (I/R-) induced mitochondrial dysfunction [74].

#### 2.1.3. MAPT

Neurons of the central nervous system are the main site of microtubule-associated protein tau (MAPT) distribution, which plays an essential role in morphogenesis, axonal transport, and axonal extension by interfering with assemblage of microtubules and stabilization of the microtubule network [75, 76]. Posttranslationally modified MAPT facilitates tubulin binding, microtubule stability, and neuronal morphology [75]. Nevertheless, if MAPT is excessively phosphorylated, the microtubule binding capacity will be reduced. As microtubules are reduced in binding capacity, the neuronal cytoskeleton becomes less stable, resulting in neuronal death [77]. Research on MAPT is mainly conducted in neurodegenerative disease pathogenesis [78]. Aggregation and hyperphosphorylation of the MAPT proteins in the brain are pathological features that exist in a large group of neurodegenerative conditions, which are named tauopathies. In addition, oxidative stress (OS) is another crucial aspect of tauopathies' pathophysiology [78].

In recent years, MAPT has gained wide attention for its potential role in stroke. Researchers have found that brain ischemia/reperfusion (CIR) animal models have high abnormally hyperphosphorylated MAPT, which is closely linked to neurological deficits and neuronal apoptosis [79]. In the research of Fujii et al., an MCAO model showed abnormally high phosphorylation of MAPT 12 hours after CIR in Wistar rats [80]. Knockout of MAPT prevented brain damage in mice after MCAO-induced stroke [81]. Several studies have demonstrated that hyperacetylation of MAPT promotes the accumulation of phosphorylated MAPT, harming cells by accumulating abnormal MAPT [77, 82]. In recent years, SIRT1 has been shown to be closely associated with MAPT modification [83, 84]. Some specific lysine residues in MAPT can be deacetylated by SIRT1, which means that a pivotal role is played by SIRT1/MAPT pathway during stroke recovery [83]. Shi et al. proved that inhibition of Sirt1/MAPT signaling by astragaloside IV (AS-IV) protects rats from cerebral ischemia/reperfusion injury. By upregulating SIRT1 expression, AS-IV decreases acetylated MAPT (ac-MAPT) and phosphorylated MAPT (p-MAPT) levels, ultimately reducing infarction size and improving neurological function [85]. However, there is no direct evidence to prove that the Sirt1/MAPT pathway plays a role in stroke directly through antioxidant responses.

#### 2.1.4. Nuclear Factor Erythroid 2-Related Factor 2 (Nrf2)

Nrf2, a basic leucine zipper protein (bZIP), is important for maintaining redox homeostasis in cells. Nrf2 is a pivotal regulator of endogenous antioxidant defenses [86], which can activate the transcription of its downstream antioxidant genes, including heme oxygenase-1 (HO-1), quinone oxidoreductase-1 (Nqo1), superoxide dismutase (SOD), catalase (CAT), and other phase II antioxidant enzymes [87, 88]. Typically, Kelch-like ECH-associated protein 1 (Keap1) retains Nrf2 in the cytoplasm. The Nrf2 protein translocates into the nucleus upon oxidative stress, binding to the antioxidant response element (ARE) and promoting antioxidant enzyme synthesis and phase II detoxification enzyme synthesis. According to recent research, neurons are protected against ischemic stroke injury by Nrf2. Knockout of the Nrf2 gene enormously increased the cerebral infarcted region and neurologic deficits in ischemia–reperfusion rats [89]. The Nrf2-target gene pathway is protective against ischemia/reperfusion injury in the brain. Increased Nrf2 activity can reduce the oxidative stress that occurs during stroke and alleviate brain injury.

Numerous regulators also control the activation of Nrf2, including SIRT1. A growing body of evidence indicates that SIRT1 plays a crucial role in regulating Nrf2. SIRT1 can deacetylate Nrf2 to increase downstream antioxidase expression. Mei et al. proved that a neuroprotective effect of diosmetin was observed both in vitro and in vivo against cerebral ischemia/reperfusion, which was mediated by inhibiting oxidative stress by regulating the SIRT1/Nrf2 signaling pathway [90]. Diosmetin induces the expression of SIRT1 and N-Nrf2, and T-Nrf2 promotes Nrf2 translocation to the nucleus and increases the expression of the downstream antioxidants NQO1 and HO-1.

### 2.2. SIRT1-Mediated Anti-inflammatory in Stroke

Inflammation plays a crucial role in stroke pathophysiology and is being targeted for stroke treatment. In human stroke cases, inflammatory cells infiltrate the brain within minutes to days after ischemic insult [91, 92], which further leads to the release of a large number of cytokines and chemokines [93]. Microglia are resident macrophages in the central nervous system. When they detect ischemia, they initiate a response immediately [94, 95, 96]. Microglial activation in the peri-infarct zone within 30 minutes to 1 hour after MCAO is accompanied by the appearance of CD11b, CD45, and Iba1 [97, 98]. At the same time, CD11b+ microglia within the infarct start fragmentation 12 hours after MCAO, and the number of microglia is reduced 24 hours later [98, 99]. There is persistent activation of microglial cells in the peri-infarct weeks after MCAO [100]. Apart from the above, infiltrating leukocytes, including polymorphonuclear leukocytes, monocytes/macrophages, and lymphocytes, also play crucial roles in ischemic stroke [101, 102, 103, 104]. Strokes caused by an ischemic stroke can induce the release of inflammatory cytokines, including IL-1*β* and IL-18 [105, 106]. An increase in inflammatory cytokines and neuroinflammation accompanies cerebral ischemia, aggravating neurodegeneration [107, 108]. Research suggests that interventions meant to reduce inflammation after cerebral ischemia can prevent brain damage from worsening.

SIRT1 is thought to play a critical role in brain protection. Several signaling pathways can be modulated by SIRT1 upon activation to affect neuroinflammation. SIRT1 plays a critical role in neuroprotection against brain ischemia through deacetylation and subsequent inhibition of p53 and nuclear factor-*κ*B-induced inflammatory and apoptotic pathways [25]. Some drugs acting on SIRT1 have shown practical neuroprotective function due to their antioxidative stress and anti-inflammatory properties. In an experiment using the middle cerebral artery occlusion (MCAO) model, salvianolic acid B (SalB), which has been proven protective against ischemic stroke in previous studies, reduces brain injury induced by ischemic stroke by activating SIRT1 to reduce apoptosis and inflammation [109]. Notably, TNF-*α* and IL-1*β* levels in brain tissue decreased following treatment with SalB. Ischemic stroke is accompanied by the production and release of proinflammatory cytokines (mainly TNF-*α* and IL-1*β*), as previously demonstrated [110]. In addition, SMND-309, a novel derivative of SalB, has been proven to inhibit reperfusion injury in rat brains by targeting the JAK2/STAT3 [111]. Kou et al. found that magnolol, by modulating the expression of SIRT1, exerts anti-inflammatory effects by decreasing the expression of IL-1*β* and TNF-*α* in brain tissue to protect the brain against cerebral ischemic injury [112]. Additionally, magnolol causes a downregulation of Ac-FOXO1, induced by the SIRT1 expression, which means that magnolol can also exert a protective effect against ischemic stroke via resistance function against oxidative stress. The SIRT1-mediated anti-inflammatory signaling pathway in stroke is shown in Figure 2.

#### 2.2.1. Nuclear Factor-*κ*B (NF-*κ*B)

The NF-*κ*B protein complex is an inducible transcription factor family that consists of five members with correlated structures, including NF-*κ*B1 (p50), NF-*κ*B2 (p52), RelA (p65), RelB, and c-Rel [113]. NF-*κ*B is widely considered a prototypical pathway that initiates inflammation, in which NF-*κ*B regulates inflammation and immunity in various ways [114]. NF-*κ*B is known to stimulate the expression of several proinflammatory genes, such as those that encode cytokines and chemokines, as well as those that regulate inflammasome activity [114, 115]. Typically, two signaling pathways, canonical and noncanonical (or alternative), are involved in activating NF-*κ*B [116]. Among them, proinflammatory cytokines such as TNF-*α* and IL-1 activate the canonical pathway, activating RelA- or cRel-containing complexes [117]. The noncanonical pathway is triggered by several TNF family cytokines (excluding TNF-*α*), leading to RelB/p52 activation [118]. Both pathways are important for immune and inflammatory response regulation. When molecules such as TNF-*α* bind to TNF receptors of different types, NF-*κ*B is activated, which further leads to subsequent activation processes [119]. To develop effective therapeutic strategies for inflammation-associated illnesses, a better understanding of the mechanisms that underlie NF-*κ*B activation and proinflammatory function is crucial.

Previous work has demonstrated that neuroinflammation mediated by NF-*κ*B contributes significantly to stroke-induced neurotoxicity [120, 121]. Several diseases are prevented by the anti-inflammatory action of SIRT1, which acts as a negative regulator of inflammation [122]. Notably, there has been extensive research on SIRT1 because it is abundantly present in brain tissue and plays a vital role in the central nervous system [123]. The interaction between SIRT1 and the RelA/p65 subunit of NF-*κ*B plays a key role in this process: RelA/p65 is negatively affected by acetylation of lysine 310 by SIRT1, resulting in decreased transcriptional activity and expression of proinflammatory genes [124]. SIRT1 deacetylation of RelA/p65 promotes the p65/p50 complex's interaction with I*κ*B-*α*. Through this association, the NF-B complex is transported back from the nucleus to the cytoplasm, thereby inactivating its activity. In a study by Deng et al., the activation of SIRT1 protected the brain after intracerebral hemorrhage by deacetylating NF-*κ*B/p65 [120]. These results suggest that inhibition of the NF-*κ*B inflammatory signaling pathway by activating SIRT1 can effectively protect brain tissue after stroke.

#### 2.2.2. High Mobility Group Box 1 (HMGB1)

HMGB1 is a protein in eukaryotic cells that repairs DNA damage and maintains genomic stability [125]. HMGB1, as a typical DAMP, induces inflammatory responses in the innate immune system due to injury or stress [126]. Inflammasome activation releases HMGB1 from glia and neurons, which activates receptors for advanced glycation end products (RAGE) and Toll-like receptor 4 (TLR-4) on target cells. An inflammatory response mediated by HMGB1 plays a role in various conditions, such as ischemia [127]. HMGB1 contains several extracellular receptors, with RAGE and TLR4 having been extensively studied and demonstrated to be true fields [128]. In addition to initiating several cellular responses, including inflammation, HMGB1 also participates in the activation of inflammation by binding with RAGE and TLR4 [129]. In neurons and glial cells, HMGB1 is actively released following activation of the inflammasome. This stimulates the activation of two PRRs, namely, TLR4 and RAGE. In previous studies, SIRT1 was shown to play a vital role in activating HMGB1/NF-*κ*B [130]. Various proinflammatory cytokines and chemokines are known to be induced by TLR4 activation, including TNF-*α*, IL-6, and IL-1*β*. Following SAH, proinflammatory cytokines can damage the surrounding neural cells and activate leukocytes, aggravating brain damage [131, 132, 133]. For HMGB1 to enter the extracellular environment and relocate to the cytoplasm, posttranslational modifications such as acetylation are critical. As HMGB1 relocates, hyperacetylation plays a critical role [134]. However, HMGB1 release is negatively regulated by SIRT1 [135]. HMGB1 is deacetylated by SIRT1 in vivo, thereby inhibiting the release of HMGB1 and the subsequent activation of inflammation [136].

#### 2.2.3. NLRP3

The NLRP3 inflammasome is part of the NLR family, which consists of NLRP3, apoptosis-associated speck-like (ASC) adapter protein, and procaspase-1 [137]. NLRP3 inflammasomes are expressed in microglia, astrocytes, and neurons [138]. By regulating IL-1*β* and IL-18 secretion, they play a role in ischemic stroke [139]. Some studies have found that NLRP3 is upregulated in ischemic brains and is expressed in microglia and endothelial cells, indicating that these cells are major sources of NLRP3 [139]. Priming signals induced by the Toll-like receptor (TLR)/nuclear factor NF-*κ*B pathway influence the transcription of NLRP3 [140]. The expression of pro-IL-1*β* and pro-IL-18 is increased by NF-kB stimuli, while the NLRP3 inflammasome activates caspase-1, which transforms inactive pro-IL-1*β* and pro-IL-18 into their active and secreted forms: IL-1*β* and IL-18. By initiating or amplifying downstream signaling pathways and driving proinflammatory responses, these cytokines cause cellular damage [141]. A previous study indicated that a lack of the NLRP3 inflammasome might enable rats to recover from cerebral injury after ischemic stroke by reducing infarcts and inflammatory responses [139]. Furthermore, neuronal cell death and behavioral deficits can be improved by inhibiting NLRP3 inflammasome activation in stroke models [139]. Importantly, several studies have confirmed that SIRT1 plays a key role in neuroprotection by inhibiting the activation of NLRP3 inflammasomes after ischemic stroke [142].

## 3. Therapeutic Effects of Natural Products Acting on SIRT1 in Stroke

Natural products are chemical compounds or substances produced by plants and microorganisms. From a particular perspective, natural products include everything produced by living things [143, 144]. There is high potential in developing new stroke treatments based on natural products [143, 145]. A natural product is typically seen as an environmentally sound, readily available resource with few adverse effects in the field [122] which makes them more clinically useful. In addition, SIRT1 plays an important role in stroke pathogenesis via its ability to modulate oxidative stress and inflammation [25]. This section is aimed at summarizing the natural products acting on SIRT1 for stroke treatment. The natural products working on SIRT1 in hemorrhagic and ischemic strokes are shown in Tables 1 and 2, respectively.

### 3.1. Natural Products Acting on SIRT1 in Hemorrhagic Stroke

#### 3.1.1. HLY78

As a novel lycorine derivative, HLY78 has shown antiapoptotic effects in tumors, ICH, and SAH [146, 147, 148]. After intranasal administration of HLY78 1 hour after ICH, it reduced oxidative stress and the extent of neuronal damage in the perihematomal region. Therefore, HLY78 may prove to be an effective drug for the treatment of ICH. Additionally, GSK3*β*/Sirt1/PGC-1*α* signaling was partially involved in the antiapoptotic and antioxidative effects [148].

#### 3.1.2. Resveratrol

Natural resveratrol is found in the skin of numerous edible plants as a stilbene polyphenol. Strokes can be treated with resveratrol by its anti-inflammatory and antioxidant effects in the field [125], which means that the neuroprotective effects of resveratrol are associated with several signaling pathways. More importantly, resveratrol is also a SIRT1 activator. Through deacetylation of p65, SIRT1 inhibits NF-*κ*B in ICH. In ICH patients, the activation of SIRT1 by resveratrol led to a neuroprotective effect and a reduction in Ac-p65, IL-1*β*, TNF-*α*, and apoptosis [120].

#### 3.1.3. Fucoxanthin (Fx)

Fx is a kind of xanthophyll derivative extensively distributed in seaweeds. This compound has an allenic bond and a 5,6 monoepoxide structure, making it a potent antioxidant. The efficacy of FX in animal models of cerebral ischemia/reperfusion injury, Alzheimer's disease, and traumatic brain injury has been demonstrated [149]. By activating Sirt1 and further deacetylating FOXO and p53, Fx has been shown to decrease oxidative damage and brain injury after SAH, indicating that Fx may act as a promising therapeutic agent for SAH [150].

#### 3.1.4. Salvianolic Acid B (SalB)

An extract of the traditional Chinese herb SalB has been shown to possess antioxidant and neuroprotective properties in vitro and in vivo [151, 152]. The central nervous system (CNS) can be directly affected by SalB because it can easily traverse the blood–brain barrier (BBB). When it is used in patients with SAH, it can reduce oxidative damage from SAH through SalB's ability to enhance SIRT1 activity and further promote Nrf2 signaling pathway activation [153].

#### 3.1.5. Melatonin

Melatonin (Mel, N-acetyl-5-methoxytryptamine), mainly secreted by the pineal gland, has shown various benefits, such as antioxidation, anti-inflammation, and antiapoptosis [154, 155, 156]. Experimental SAH models have shown Mel to be protective, reducing mortality after a severe subarachnoid hemorrhage [157]. A subsequent experiment further confirmed that the MR/Sirt1/NF-*κ*B pathway is activated by Mel and reduces apoptosis following SAH [158].

#### 3.1.6. Berberine

Berberine is an isoquinoline alkaloid found in the Chinese herb Coptis chinensis that has anti-inflammatory and neuroprotective properties. The activation of HMGB1/NF-*κ*B plays a crucial role in cerebral inflammation in SAH [159]. The interaction between HMGB1 and TLR4 triggers inflammatory responses after SAH insults. Following TLR4 activation, NF-*κ*B is active, and proinflammatory cytokines and chemokines are released [160]. Inflammatory responses mediated by HMGB1/NF-*κ*B activation can be inhibited by berberine supplementation by increasing the expression of SIRT1 [161].

#### 3.1.7. Oleanolic Acid (OA)

OA (3b-hydroxy-olea-12-en-28-oic acid) is a triterpenoid compound that comes from various sources and can reduce inflammation and enhance antioxidant activity. Upon inflammasome activation, neurons and glia release HMGB1, which activates the RAGE receptor on target cells and the TLR4 receptor in the immune system. When OA is applied to patients with SAH, it can reduce acetylation of HMGB1 by activating SIRT1 to alleviate early brain injury after subarachnoid hemorrhage, which has been demonstrated to exert neuroprotective effects through its anti-inflammatory role [162].

#### 3.1.8. Carnosic Acid (CA)

The CA is one of the most abundant phenolic compounds in rosemary and sage leaves, exhibiting antioxidant and antiapoptotic properties [163]. In a study, CA was applied to a vascular perforation model, which was used to mimic clinical SAH, and the desired therapeutic effect was obtained. There was a dramatic reduction in neuronal cell death and brain edema with CA treatment in ICH, as well as a diminished level of ROS [164]. The SIRT1/p66shc pathway may play a role in the protective effect of CA on SAH.

#### 3.1.9. Wogonoside

The herb Scutellaria belongs to the Labiatae family (containing approximately 400 species) and is used for treating inflammation, allergies, and hepatitis, and as an antioxidant. A compound isolated from Scutellaria called wogonin is a radical scavenger, an anticancer agent, and an antioxidant [165]. When wogonoside is used in SAH treatment, it activates SIRT1 and decreases the level of p53 to prevent neuronal apoptosis [166], mainly through its anti-inflammatory properties.

#### 3.1.10. Piceatannol (Pic)

A hydroxylated analog of resveratrol called Pic has proven to be anti-inflammatory and potent antioxidant properties. A major mechanism through which Pic exerts its antioxidant effects is by upregulating antioxidant enzymes, such as SOD and CAT [167]. There was a dose-dependent increase in antioxidant activity and suppression of apoptosis with Pic, as well as upregulation of Sirt1/FoxO1 signaling in stroke [168]. It proved that Pic potentially exerts neuroprotective effects through upregulation of Sirt1/FoxO1 signaling in stroke.

### 3.2. Natural Products Acting on SIRT1 in Ischemic Stroke

#### 3.2.1. Adiponectin (APN)

APN, which is entirely released by adipocytes, has been proven to act as a neuroprotectant in ischemia/reperfusion injuries [169, 170]. Past research suggested that there is an important role played by glutamate- (Glu-) induced excitotoxicity in stroke. When APN was used in HT22 neurons of Glu-induced injury, it upregulated the SIRT1, PGC-1*α*, and SOD. It downregulated the ROS levels, which suggested that the APN peptide activates PGC-1*α* signaling in HT22 neurons in response to Glu-induced injury [53].

#### 3.2.2. Salvianolic Acid B

In addition to having a role in the SAH model, SalB is also protective against ischemic stroke. The expression of SIRT1 and Bcl-2 was upregulated by SalB in the MCAO model, while the expression of Ac-FOXO1 and Bax was downregulated. SalB treatment exerts cerebroprotective effects by reducing neuroinflammatory conditions and oxidative stress levels by activating SIRT1 signaling [109].

#### 3.2.3. Alpha-Lipoic Acid (ALA)

The ALA is derived from octanoic acid, which acts as a cofactor in several mitochondrial dehydrogenases [171]. As an active free-radical scavenger, ALA exhibits powerful antioxidative properties [172]. After the systemic administration of ALA, SIRT1 and PGC-1*α* expressions were significantly increased, indicating the activation of SIRT1/PGC-1*α* might contribute to its beneficial effect.

#### 3.2.4. Astragaloside IV (AS-IV)

For more than a thousand years, Astragalus membranaceus root and Mongolian Astragalus powder have been used to treat ischemic stroke [173], of which AS-IV is the predominant active component. The anti-inflammatory and antioxidative properties of AS-IV have been demonstrated in previous studies [174, 175]. In an earlier study, AS-IV contributed to the decrease in infarction area and the improvement of neurological functions. Additionally, the level of SIRT1 expression was upregulated, and ac-MAPT and p-MAPT declined [85]. Thus, the Sirt1/Mapt pathway is recognized to play a role in AS-IV's neuroprotective effect in rat models of CIR injury.

#### 3.2.5. Arctigenin (ARC)

One of the most abundant and bioactive compounds in ARC has several pharmacological effects, including anti-inflammation, antiapoptosis, and antitumor effects [176]. It was demonstrated that ARC treatment could effectively suppress SIRT1-driven NLRP3 inflammasome activation by ischemic stroke in rat models [142]. In the light of this finding, ARC may play an important role in attenuating the damage to the brain caused by ischemic stroke.

#### 3.2.6. Quercetin

A natural flavonoid, quercetin, is found in rutin and various fruits and vegetables. Quercetin is a potent ROS scavenger and has been shown to positively affect BBB function in acute ischemic strokes due to its ability to scavenge ROS. In research on the MCAO rat model, quercetin treatment was identified to suppress oxidative stress by activating Sirt1/Nrf2/HO-1 signaling pathways [177].

#### 3.2.7. Momordica charantia Polysaccharides (MCPs)

MCPs, the main practical component extracted from Momordica charantia (MC), can protect against nerve damage after stroke by scavenging free radicals [178]. Under glutamate injury, MCPs activate SIRT1, improving the nuclear accumulation of *β*-catenin and contributing to NSC differentiation into neurons in the mimic IRI cell model [179]. Considering this study's findings, MCPs may protect patients recovering from ischemic stroke at late stages.

#### 3.2.8. Icariin (ICA)

ICA is an active flavonoid with antioxidative and immunoregulatory effects. After MCAO, ICA has been shown to significantly attenuate brain damage, with the mechanism being an elevation of PGC-1*α*, which depends on SIRT1 [180]. It is, therefore, possible to develop ICA as a neuroprotectant for ischemia-related brain damage.

#### 3.2.9. Kaempferol (KFL)

KFL is a natural product obtained from several natural sources that possesses antioxidative and immunoregulatory properties [181]. A cell model of ischemia/reperfusion injury showed that KFL effectively prevented OGD-induced cytotoxicity. The protection provided by KFL depends on the expression of SIRT1 and the inhibition of P66shc expression and acetylation [182].

#### 3.2.10. CG

CG is a calycosin derivative compound derived from Astragali Radix (RA) and a representative component of isoflavones in RA. A significant improvement in cell viability and a reduction in neuronal apoptosis were observed with CG in the ischemia-reperfusion model in vitro. Additionally, CG treatment increased the expression of SIRT1, FOXO1, PGC-1*α*, and Bcl-2 while decreasing the expression of Bax [58]. This implies that GC exerts its neuroprotective role through activating SIRT1/FOXO1/PGC-1*α* signaling.

#### 3.2.11. Notoginseng Leaf Triterpenes (PNGL)

PNGL are isolated from Panax notoginseng (Burk) and purified as a medicinal resource, functional, and typical food. Some studies have indicated that the neuronal apoptosis induced by ischemia is attenuated by PNGL, exerting potent neuroprotective effects. PNG exerts its protective effects via the NAMPT-NAD+ pathway and downstream SIRT1/2/3-Foxo3a-MnSOD/PGC-1*α* pathways [183].

#### 3.2.12. Cycloastragenol (CAG)

CAG, an aglycone of astragaloside IV, was detected when looking for antiaging active ingredients in Astragalus membranaceus extracts [184]. It was found that a dose-dependent decrease in brain infarct volume was observed with CAG, as well as significant improvements in functional deficits and a decrease in neuronal loss in MCAO mice treated with CAG [185]. Its beneficial effect involves upregulating SIRT1, thereby inhibiting neuroinflammation.

## 4. Conclusion and Perspectives

Strokes are cerebral vascular diseases with a high mortality rate, deadly cerebral vascular disorders with a high mortality rate, and substantial economic and social costs. A stroke can be classified as either an ischemic stroke or a hemorrhagic stroke. Regardless of the type of stroke, however, oxidative stress and neuroinflammation have been linked to the subsequent brain injury and play vital roles. Accordingly, the treatment that reduces oxidative damage and inflammation after stroke to improve neurological recovery has long been a focus of stroke treatment research. SIRT1, as an NAD-dependent deacetylase in the nucleus, has been proven to play a critical role in oxidative stress and neuroinflammation in stroke. SIRT1 modulates oxidative stress and inflammation through a variety of signaling pathways. Therefore, a comprehensive understanding of the signaling pathway in the process of SIRT1-mediated antioxidation and anti-neuroinflammation in stroke is fundamental and can be used as the basis for therapies in stroke. At the same time, due to its numerous merits, such as readily available resources and few adverse effects, natural products have excellent application and practical clinical value in treating stroke. There are, however, some limitations to our literature review. Studies of natural compounds with possible neuroprotective effects in stroke are still in the exploratory stage, and clinical studies have yet to be conducted. This review discusses the potential mechanisms and natural products used in stroke by which Sirt1 protects against stroke through antioxidative and anti-inflammatory effects. It has considerable significance for future approaches to improving stroke treatment.

## Figures and Tables

**Figure 1:** The signal pathway of SIRT1-mediated antioxidation in stroke. The picture shows the signal pathway of SIRT1-mediated antioxidation in stroke. In response to oxidative stress after stroke, SIRT1 mainly mediates four molecular modifications, including Nrf2, FOXO, PGC-1*α*, and MAPT. By deacetylating the major acetylation sites, the level of FOXO, PGC-1*α*, and Nrf2 is upregulated by SIRT1, while MAPT is downregulated. When the level of FOXO, PGC-1*α*, and Nrf2 increases, several kinds of antioxidant proteins also correspondingly increase, which further suppress oxidative stress. In addition, the accumulation of abnormal MAPT will be reduced through deacetylating MAPT, thus reducing the damaging effect on cells. Therefore, some drugs or upstream regulators can inhibit oxidative stress by acting on SIRT1, which further exerts neuroprotective effects.

**Figure 2:** The signal pathway of SIRT1-mediated anti-inflammatory in stroke. The picture shows the signal pathway of SIRT1-mediated anti-inflammatory in stroke. SIRT1 can inhibit the production of proinflammatory factors through the deacetylation of HMGB1, NF-*κ*B, and NLRP3 inflammasome, thus achieving an anti-neuroinflammatory effect. Through the deacetylation of HMGB1 and NF-*κ*B, the synthesis of some proinflammatory cytokines such as TNF-*α*, IL-6, and IL-1*β* in the nucleus was inhibited. In addition, through the deacetylation of the NLRP3 inflammasome, the function of caspase-1 was restricted, and eventually, the pathway of conversion of pro-IL-1*β* and pro-IL-18 to IL-1*β* and IL-18 was blocked.

**Table 1:** The natural products acting on SIRT1 in hemorrhagic stroke.

Studied drugs	Mechanisms	Classes of action	Animal models	Reference
HLY78	GSK3*β*/Sirt1/PGC-1*α* pathway	Antioxidation	ICH model (induced via autologous blood injection)	Jin et al. [148]
Resveratrol	NF-*κ*B/p65 deacetylating	Anti-neuroinflammation	ICH model (intracranial injection of type IV collagenase)	Deng et al. [120]
Fucoxanthin (Fx)	Activating Sirt1 and further deacetylating FOXO and p53	Antioxidation	SAH model (prechiasmatic cistern injection models)	Zhang et al. [150]
Salvianolic acid B (SalB)	Activating SIRT1 and Nrf2 signaling pathway	Antioxidation	SAH model (single blood injection)	Zhang et al. [153]
Melatonin (Mel)	Activating MR/Sirt1/NF-*κ*B pathway	Anti-neuroinflammation and antioxidation	SAH model (endovascular perforation model)	Zhao et al. [158]
Berberine	Activating sirtuin 1 and suppressing HMGB1/NF-*κ*B pathway	Anti-neuroinflammation	SAH model (prechiasmatic cistern injection models)	Zhang et al. [161]
Oleanolic acid	SIRT1-mediated HMGB1 deacetylation	Anti-neuroinflammation	SAH model (endovascular perforation model)	Han et al. [162]
Carnosic acid (CA)	Activating SIRT1/p66shc pathway	Antioxidation	SAH model (endovascular perforation model)	Teng et al. [164]
Wogonoside	Activating SIRT1 and further deregulating p53	Anti-neuroinflammation	SAH model (endovascular perforation model)	Cheng et al. [166]

**Table 2:** The natural products acting on SIRT1 in hemorrhagic stroke.

Studied drugs	Mechanisms	Classes of action	Animal models	Reference
Adiponectin (APN)	Activating SIRT1/PGC-1*α*	Antioxidation	Glutamate- (Glu-) induced excitotoxicity in mouse HT22 hippocampal cells	Yue et al. [53]
Salvianolic acid B (SalB)	Downregulation of Ac-FOXO1	Anti-neuroinflammation and antioxidation	Middle cerebral artery occlusion (MCAO) model	Lv et al. [109]
Alpha-lipoic acid	Activating SIRT1/PGC-1*α* pathway	Antioxidation	MCAO	Fu et al. [186]
Astragaloside IV (AS-IV)	Activating Sirt1/Mapt pathway	Antioxidation	MCAO	Shi et al. [85]
Arctigenin (ARC)	NLRP3 inflammasome	Anti-neuroinflammation	MCAO	Zhang et al. [142]
Quercetin	Activating SIRT1/Nrf2 pathway	Antioxidation	MCAO	Yang et al. [177]
Momordica charantia polysaccharides (MCPs)	Activating SIRT1/*β*-catenin pathway	Antioxidation	MCAO	Hu et al. [179]
Icariin (ICA)	Activating SIRT1/PGC-1*α* pathway	Antioxidation	MCAO	Zhu et al. [180]
Kaempferol (KFL)	Activating SIRT1/P66shc pathway	Antioxidation	Oxygen and glucose deprivation (OGD)	Zhou and Li [182]
Calycosin-7-O-*β*-D-glucoside (CG)	Activating SIRT1/FOXO1/PGC-1*α* pathway	Antioxidation	OGD	Yan et al. [58]
Notoginseng leaf triterpenes (PNGL)	Activating SIRT1/2/3-Foxo3a-MnSOD/PGC-1*α* pathways	Antioxidation	OGD	Xie et al. [183]
Cycloastragenol (CAG)	Suppression of SIRT1/NF-*κ*B activation	Anti-neuroinflammation	MCAO	Li et al. [185]
Piceatannol	Activating Sirt1/FoxO1 pathway	Antioxidation	MCAO	Wang et al. [168]

## Data Availability

No data were used to support this study.
